The article "Treatment with Panax Ginseng Antagonizes the Estrogen Decline in Ovariectomized Mice" was retracted in 2020. Reasons: duplicated images; concerns about the data.

# Treatment with Panax Ginseng Antagonizes the Estrogen Decline in Ovariectomized Mice

**DOI:** 10.3390/ijms15057827

**Published:** 2014-05-06

**Authors:** Ying Xu, Jie Ding, Xiao-Ping Ma, Ying-Hui Ma, Zhi-Qiang Liu, Na Lin

**Affiliations:** 1 Institute of Chinese Materia Medica, China Academy of Chinese Medical Sciences, Dongcheng District, Dongzhimen Nanxiao Road 16, Beijing 100700, China; E-Mails: xu_ying1978@163.com (Y.X.); dingjie135@163.com (J.D.); ma_yy_6669@163.com (X.-P.M.); 2 Changchun Institute of Applied Chemistry, Chinese Academy of Sciences, Renmin Road 5625, Changchun 130022, China; E-Mails: myh0131@sohu.com (Y.-H.M.); liuzq@ciac.jl.cn (Z.-Q.L.)

**Keywords:** ginseng, estrogenic activity, uterus, vagina, ER α, ER β

## Abstract

Ginseng is a popular herb for alleviating menopausal symptoms; however, no conclusive scientific data has shown ginseng as being efficient in such therapies. The present study was designed to evaluate the estrogenic efficacy of ginseng on reproductive target tissues of ovariectomized (OVX) mice. The OVX mice were treated with ginseng at doses of 12.0, 18.0 and 24.0 g/kg per day for four weeks. Ginseng treatments restored the estrus cycle and demonstrated significant estrogenic activity, as indicated by the reversal of the atrophy of the uterus and vagina, upregulation of estrogen receptor (ER) α and ER β expression at the protein and mRNA level in the reproductive tissues, where ER α upregulation was stronger than that of ER β. Meanwhile, treatment with ginseng significantly increased adrenal gland weight and serum estradiol and clearly decreased follicle-stimulating hormone (FSH) and luteinizing hormone (LH) in circulation. Notably, the largest changes in these parameters were found at the highest dose of 24.0 g/kg. Moreover, ginseng at 18.0 g/kg resulted in the greatest decrease in weight gain caused by ovariectomy. The data suggest that ginseng estrogenic responses show tissue variation that reflects different affinities of ERs for ginseng components. This study demonstrates that ginseng activity is mediated through estrogenic components and provides further evidence for ginseng treatment of postmenopausal symptoms.

## 1. Introduction

Ginseng is a popular herbal medicine that has been used for over 2000 years in oriental countries. It has been reported that ginseng has a wide range of pharmacological activities in the cardiovascular, endocrine, immune and central nervous systems [1]. Studies have shown that ginseng could relieve menopausal symptoms, bleeding disorders, sleeping disorders, depression and anxiety [2–4], which indicating that some components of ginseng act as phytoestrogens and/or involve the activation of the estrogen receptor (ER) [5]. *In vitro* studies also have shown that ginseng extracts are able to stimulate the growth of ER-positive cells [6]. Ginsenoside-Rg_1_, -Rb_1_ and -Rh_1_ have been shown to contain estrogen-like activity and activated the ER [7–9]. However, despite ginseng being a popular herb for the alleviation of menopausal symptoms and extensively used as an alternative for hormone replacement therapy, no conclusive scientific data has shown that ginseng is efficient in such therapies, in contrast to the extensive studies on the estrogenic activity of isoflavones found in soybeans [10]. It is clear that the efficacy and molecular mechanisms of ginseng need to be elucidated for safer use of this promising therapy. The purpose of this study was to investigate the *in vivo* estrogenic properties of ginseng used by ovariectomized (OVX) mice. This is the first *in vivo* study to evaluate the estrogenic efficacy of ginseng on reproductive target tissues of OVX mice. However, it should be pointed out that this is very likely not the only pathway of ginseng action. In the present study, we aimed to characterize the estrogenic effects of ginseng on ovariectomized mice by observing estrous cycle, body weight gain, hormone level, measuring the histologic structure changes and estrogen receptors (ER α and ER β) expression in reproductive target tissues, as part of an ongoing effort to provide scientific data on ginseng and to identify potent agents for the prevention and treatment of postmenopausal syndrome.

The article "Treatment with Panax Ginseng Antagonizes the Estrogen Decline in Ovariectomized Mice" was retracted in 2020. Reasons: duplicated images; concerns about the data.

## 2. Results

### 2.1. Analysis of Water Extract of Panax Ginseng

The ginseng extract used in this trial contained 0.228% of Rb_1_, 0.252% of Rf, 0.252% of Rc, 0.636% of Rg_2_, 0.06% of Rd and 0.456% of Rg_1_ and Re. The total ginsenosides, calculated as the sum of the above individual ginsenosides, represented 1.884% in the ginseng extract. The chromatogram of the ginseng extract is presented in Figure 1.

### 2.2. Effect of Ginseng on the Estrus Cycle

To characterize the estrogenic activity of ginseng on the reproductive tissue of OVX mice, we compared the activity with a synthetic estrogen, estradiol valerate. The estrous cycle of all mice was monitored by daily inspection of vaginal epithelium cell smears. As shown in Figure 2i, smears of the vaginal epithelium cells from OVX mice consisted of leukocytes, which is indicative of constant diestrus; the estrous cycle of none of the mice in this group was restored during the period of administration. In contrast, the vaginal cells from the OVX mice treated with ginseng (12.0, 18.0 or 24.0 g/kg) or estradiol valerate became keratinized after treatment for about seven days, indicating that the status of estrus in the OVX mice was restored (Figure 2ii,iii). All of the sham-operated mice gradually restored the estrous cycle (not shown). Moreover, treatment with ginseng prolonged the estrous stage of the OVX mice, suggesting very potent estrogenic activity.

The article "Treatment with Panax Ginseng Antagonizes the Estrogen Decline in Ovariectomized Mice" was retracted in 2020. Reasons: duplicated images; concerns about the data.

Vaginal epithelium cell smears were taken at the seventh day from ovariectomized (OVX) mice untreated (i), treated with estradiol valerate (EV) (ii) or treated with ginseng (GS) (iii). Smears from untreated OVX mice consisted of leukocytes, confirming a state of diestrus. Smears from OVX mice treated with GS or estradiol valerate showed a large number of keratinized epithelial cells, indicating that both GS and estradiol valerate can restore the estrous cycle of OVX mice.

### 2.3. Effect of Ginseng on Body, Uterine and Adrenal Gland Weights

The mice from all six groups had similar initial mean body weights. At the end of the study, the mean body weight of mice in the OVX group was significantly higher than that of the sham group. Estradiol valerate treatment completely prevented the increase in body weight associated with E_2_ deficiency from the second postoperative week (Figure 3A). Ginseng at higher dose treatment had significant effects on body weight gain, and ginseng at 18.0 g/kg resulted in the largest decrease compared with untreated controls at the fourth week (*p* < 0.001). The results suggest that ginseng could decrease body weight gain in postmenopausal women and had a better ability compared to estradiol valerate to reverse the body weight gain caused by ovariectomy.

As expected, the mean uterine weight of OVX animals was significantly lower than that of sham controls; estradiol valerate treatment significantly increased the uterine weight of OVX mice (*p* < 0.001). Treatment of OVX mice with ginseng had modest stimulatory effects on uterine weight; the higher dose (18.0 or 24.0 g/kg) treatment resulted in significant differences (both *p* < 0.05), with the largest change being a 1.9-fold increase in weight compared with untreated OVX mice. Ginseng at 18.0 or 24.0 g/kg significantly increased the adrenal gland weight of OVX mice in a dose-dependence manner, and the highest dose of 24.0 g/kg induced a 16% increase in the adrenal gland of OVX mice, which was comparable to the sham control (Figure 3B).

### 2.4. Effect of Ginseng on Levels of Serum E_2_, Luteinizing Hormone and Follicle-Stimulating Hormone

Ovariectomy is expected to lower the levels of serum E_2_ and increase the levels of Luteinizing Hormone (LH) and Follicle-Stimulating Hormone (FSH) compared with sham-operated mice. The ginseng 18.0 or 24.0 g/kg treatment of OVX mice significantly raised the levels of circulating E_2_. Ginseng at 24.0 g/kg induced a 38% increase in the E_2_ level compared to that of OVX mice, which was comparable to the sham control (Figure 4A). Ginseng treatment of OVX mice had significant stimulatory effects on LH and FSH (Figure 4B,C). There was a trend of this decreasing with an increasing dose of ginseng; the highest dose, 24.0 g/kg, resulted in a 43% decrease in LH and FSH (both *p* < 0.01) compared with untreated OVX controls, respectively.

The article "Treatment with Panax Ginseng Antagonizes the Estrogen Decline in Ovariectomized Mice" was retracted in 2020. Reasons: duplicated images; concerns about the data.

### 2.5. Effects of Ginseng on the Histology of Uterus and Vagina

Histological analysis of uterine sections revealed significant atrophy in the uterus of untreated OVX mice compared with sham controls, as indicated by obvious degeneration of the cavities, endometrium and secretory glands. Treatment of OVX mice with estradiol valerate or ginseng at 18.0 or 24.0 g/kg substantially restored uterine morphology, as indicated by the thickening of the uterine endometrium, the increased number of glands and more extended glandular cavities compared with untreated OVX samples. Thus, ginseng had a similar ability as estradiol valerate to reverse the atrophy caused by ovariectomy.

Figure 5 shows microscopic preparations of representative vagina from one animal per treatment group; compared with sham mice, the vaginal epithelium of OVX mice was atrophic, as indicated by less cell layers being present, and these were composed of flattened cells with no cornification. The estradiol valerate animals displayed typical squamous multilayered epithelium layers with cornification. Treatment with ginseng at the three doses increased epithelial thickness and also the number of cell layers.

Taken together, these studies provide evidence that ginseng has significant estrogenic activity, comparable to that of the synthetic estrogen, estradiol valerate. These data prompted further studies to elucidate the molecular basis of ginseng activity, in particular to provide evidence that the effects of ginseng are mediated through the activation of estrogen receptors (ERs).

### 2.6. Effects of Ginseng on Expression of ER Subtype in Uterus and Vagina

Representative sections of the expressions of ER α and ER β in the uterus and vagina from each group and quantitative analysis are shown in Figure 6. The expression of ER α and ER β in the uterus and vagina of untreated OVX mice were significantly decreased compared with the sham group, respectively (all *p* < 0.001), and treatment with either estradiol valerate or ginseng at the three doses induced clear and comparable upregulations of ER α and ER β, and the largest increases of them were found in the highest dose of 24.0 g/kg among the ginseng treatment groups. ERs in uterus were expressed in similar cell types in the ginseng-treated, estradiol valerate-treated or sham operated groups, namely in the epithelial cells of the endometrium, interstitial cells and smooth muscle cells. ERs in vagina were expressed in vaginal epithelium cells of squamous cell and smooth muscle cells. These data further support the indication that ginseng mediates its activity *in vivo* through ERs.

The article "Treatment with Panax Ginseng Antagonizes the Estrogen Decline in Ovariectomized Mice" was retracted in 2020. Reasons: duplicated images; concerns about the data.

### 2.7. Effect of Ginseng on Protein and Gene Levels of ER Subtype in Uterus and Vagina

Further evidence for the interaction of the ginseng with the ER system was sought by determining the effects on ER subtype expressions on protein and mRNA levels in target tissues by western blot and real-time quantitative PCR. The results, as shown in Figure 7A,B, compared with the sham group, demonstrate that both protein and gene expression of ER α and ER β was significantly decreased in the uterus and vagina of OVX mice (all *p* < 0.001). Treatment with either estradiol valerate or ginseng at the three doses induced significant upregulations of ER α and ER β on protein and mRNA levels in target tissues. The highest dose, 24.0 g/kg, resulted in the largest upregulation of protein expression with 2.95-fold in ER α (*p* < 0.001) and 2.55-fold in ER β (*p* < 0.001) in the uterus, respectively, compared with untreated OVX mice. Ginseng at 24.0 g/kg also upregulated 2.98-fold ER α (*p* < 0.001) and 2.48-fold ER β (*p* < 0.001) in vagina. Meanwhile, compared with untreated OVX mice, the effects of ginseng and estradiol valerate on the gene expression of ER α and ER β in target tissue were similar to those in protein levels.

## 3. Discussion

In view of phytoestrogens being similar both structurally and functionally to mammalian estrogens, but with reportedly lower side effects compared with synthetic estrogen, therefore, seeking effective phytoestrogens is an important and urgent issue in the prevention and treatment of postmenopausal syndrome. Ginseng has been a popular herbal medicine for the alleviation of menopausal symptoms and was extensively used as an alternative for hormone replacement therapy. However, no conclusive scientific data has shown that ginseng is efficient in such therapies. In the present study, we evaluated the estrogenic activity of ginseng on an ovariectomized mice model. The results showed that ginseng has a potent estrogenic activity on OVX mice, as indicated by the restoration of the estrus cycle, antagonizing target tissue atrophy and estrogen decline in circulation caused by ovariectomy. In addition, ginseng could relieve the symptom of weight increase induced by estrogen decline. Ginseng’s estrogenic activity may be mediated by stimulating the biosynthesis of estrogen and increasing the quantity of ERs in the target organs.

The article "Treatment with Panax Ginseng Antagonizes the Estrogen Decline in Ovariectomized Mice" was retracted in 2020. Reasons: duplicated images; concerns about the data.

Estradiol-17β (E_2_), a reproductive hormone, plays a vital role in body weight control [11]. In postmenopausal women, estrogen deficiency is associated with the increased probability of obesity [12]. Consistently, ovariectomized mice deficient for estrogen that are developing obesity can have the obesity reversed by E_2_ replacement therapy, which can be achieved by decreasing food intake and increasing energy expenditure [13]. Importantly, experimental data *in vivo* and *in vitro* have provided evidence that estrogen signaling modulates fat accumulation and body weight by binding to ER α [14–18]. Our data showed that ginseng as a phytoestrogen also profoundly inhibited body weight increase and upregulated the expression of ER α in the target tissue of OVX mice.

Estrogens are synthesized in the ovary or testis and adrenal gland [17]. The adrenal gland becomes the principal tissue for secreting estrogen after ovariectomy. The increased weight of adrenal gland and serum estrogen concentration after treatment with ginseng suggests that at higher doses, the effect of ginseng may be mediated through the hypothalamus-pituitary-adrenal axis and stimulate the biosynthesis of estrogen in the adrenal gland. Using LH serum levels as a marker of estrogenic effect in the hypothalamus, where the gonadotropin-releasing hormone pulse generator resides [18], ginseng seems to be effective in reducing the activity of this brain structure.

Under physiological conditions, the biological effects of estrogen depend on not only the level of estrogen, but also on the distribution and expression levels of the corresponding ERs in the target cell, ER α and ER β [19–21]. Estrogen and ERs are involved in the physiological function and regulation of the female reproductive system. In our present study, ginseng significantly upregulated the expressions of ER α and ER β in protein and gene levels in the target tissues, respectively. It is worth mentioning that ER α upregulation induced by ginseng extract was stronger than that of ER β, suggesting that ginseng may bind to ER α with higher selectivity than ER β in reproductive target tissues.

Ginsenosides, especially their aglycone part, are similar to several steroids in structure, including female hormones, so they have been shown to possess estrogen-like activities. In a recent report [10,22], Ginsenosides showed two types of regulatory effect on ERs: Rg_1_ acted as ER α-selective agonists and, only at a high concentration, activated ER β; whereas Rb_1_ activated both ER α and ER β. It is likely that the ability of ginseng to upregulate both ERs can be explained by the presence of multiple active components contained in the herb’s ingredients, which together exhibit polyvalent activities on ER regulation in target tissue. Chen *et al.* reported [23] that chronic administration of ginsenoside Rg_1_ did not result in any estrogenic effects on reproductive tissues in an OVX animal model, which suggests that other components in ginseng exert activity on reproductive target tissues. Shim *et al.* reported [24] that chronic administration of 2 g/kg ginseng extract did not result in uterine weight increase in an OVX rat. Meanwhile, our preliminary experiment results demonstrate that treatment of immature mice with ginseng intragastrically at a daily dose of 0.5, 1.0, 1.5, 3.0 and 6.0 g/kg also did not result in the increasing of uterine weight and the raising of the E_2_ level in circulation, which suggests that the low dosage of ginseng may have resulted in no effectiveness.

The article "Treatment with Panax Ginseng Antagonizes the Estrogen Decline in Ovariectomized Mice" was retracted in 2020. Reasons: duplicated images; concerns about the data.

## 4. Experimental Section

### 4.1. Herbal Preparation and Analysis

Radix ginseng was purchased from Changchun Medicinal Herbs Co., Ltd. (Jilin, China) and identified and authenticated by an expert at the Changchun Institute of Applied Chemistry, Chinese Academy of Sciences. Radix ginseng was pulverized to a fine powder and boiled twice with distilled water for 1 h under reflux. The aqueous extracts were collected and filtered. The filtrates were then concentrated under reduced pressure at 50 °C and to a concentration of 0.6 g/mL. An high performance liquid chromatography (HPLC) method was developed for the quantification of ginsenosides in the ginseng extract. The HPLC system used was a Waters 2695 equipped with a UV detector at 210 nm. The stationary phase used was a Kromasil C18 column (5 μm, 4.6 mm × 250 mm, Akzo Nobel, Amsterdam, The Netherlands) thermostated at 25 °C. The mobile phases were acetonitrile (25%~50%) (Fisher, Waltham, MA, USA) and water (75%~50%) (Milli-Q, Boston, MA, USA) running at 0.8 mL/min for 55 min.

### 4.2. Animals and Treatment

Four-week-old female Kunming (KM) mice (Experimental Animal Center of Academy of Military Medical Sciences, Beijing, China) maintained normal 5-day estrous cycles as confirmed by daily vaginal epithelium cell smear testing until the ovariectomy was performed. The dorsal ovariectomy was performed under general anesthesia using 30 mg/kg of pentobarbital and 500 mg/kg urethane. All ovariectomized mice were checked by daily vaginal epithelium cell smear analysis, in which 5 consecutive days of leukocytes were indicative of constant diestrus and successful ovariectomy. In sham-operated negative controls, fat near the ovary was removed. The mice were randomly assigned to six groups: ovariectomized without treatment (OVX, *n* = 10), sham operated (sham, *n* = 10), ovariectomized mice treated with 0.154 mg/kg estradiol valerate (EV, *n* = 10) and OVX mice treated with ginseng intragastrically at a daily dose of 12.0, 18.0 or 24.0 g/kg per day for 4 weeks. Dose calculations followed the guidelines correlating dose equivalents between humans and laboratory animals, on the basis of the ratios of body surface area; 0.15~1.5 g/kg is the recommended dose in humans. Untreated control ovariectomized mice and sham mice received distilled water only. All animals were maintained on a 12-h light/dark cycle under constant temperature (24 ± 2 °C) and humidity (55% ± 5%) and allowed free access to food and water. All procedures for consideration of animal welfare were reviewed and approved by the ethical committee of China Academy of Traditional Chinese Medicine in April 2013 (the project identification code: 2013-58).

The article "Treatment with Panax Ginseng Antagonizes the Estrogen Decline in Ovariectomized Mice" was retracted in 2020. Reasons: duplicated images; concerns about the data.

### 4.3. Monitoring Estrus Cycle

All mice were monitored by daily vaginal epithelium cells smear testing during the 4-week administration period. The vaginal lavage was fixed with 95% ethanol for 10 min and stained with methylene blue for 10 min [25]. Vaginal epidermal cells were observed by microscopy, and keratinized vaginal cells were taken as being indicative of estrus.

### 4.4. Analysis of Tissue and Serum

Animals were sacrificed by decapitation after 8 weeks of treatment. Blood was collected from the retro-orbital plexus for analysis of E_2_, FSH and LH by enzyme linked immunosorbent assay (ELISA). The uterus and adrenal gland were removed and weighed. The left horns of the uterus and vagina were stored at −80 °C, and the right horns of the uterus and the rest of vagina were fixed with 4% polyoxymethylene for 24 h. All samples were embedded in paraffin and prepared for cross-sections; sections 4 mm-thick were cut, mounted and stained with hematoxylin and eosin (H&E) for microscopy.

### 4.5. Immunohistochemistry

Tissue sections 4 mm-thick of uterus and vagina were mounted on polylysine-coated slides. The paraffin sections were dewaxed by a routine method and incubated for 10 min with 3% hydrogen peroxide (H_2_O_2_). Each section was incubated with blocking serum (Vectastain ABC Kit, Vector Laboratories Ltd., Burlingame, CA, USA) at room temperature for 30 min and then with primary rabbit anti-estrogen receptor-α antibody (dilution 1/30, Abcam Biotechnology, Abcom Ltd., Cambridge, UK) and a rabbit anti-estrogen receptor-β (dilution 1/30, Abcam Biotechnology), respectively, overnight at 4 °C. Sections incubated in phosphate-buffered saline (PBS) without antibody served as negative controls. After incubation with biotinylated secondary antibody, sections were incubated with an avidin-biotin complex reagent containing horseradish peroxidase for 30 min. The sections were then stained with 3,3′-diaminobenzidine (DAB) (Sigma, Sigma-Aldrich Company, St. Louis, MO, USA) [26]. The Image-Pro Plus 6.0 System image analysis system was used for quantitative analysis.

The article "Treatment with Panax Ginseng Antagonizes the Estrogen Decline in Ovariectomized Mice" was retracted in 2020. Reasons: duplicated images; concerns about the data.

### 4.6. Western Blot

Uterus and vagina were resuspended in lysis buffer (50 mM Tris, pH 8.0, 150 mM NaCl, 5 mM EDTA, 0.1% sodium dodecyl sulfate (SDS), 0.5% NP-40) containing 10 mM phenylmethylsulfonyl fluoride (PMSF) and 2 mg/mL aprotinin. The protein was obtained to detect the levels of ER α and ER β in target tissue by western blot. The western blot protocol and semi-quantitative analysis were carried out as described [27]. The antibody of rabbit anti-ER α polyclonal antibody (dilution 1/100, Abcam Biotechnology) or mouse anti-ER β monoclonal antibody (dilution 1/1,000, Abcam Biotechnology) was used. All experiments were done in triplicate. The relative quantity of each antibody was measured by Alpha Ease FC (Fluorchem FC_2_) software. The density ratio of protein to glyceraldehyde 3-phosphate dehydrogenase (GAPDH) was calculated from the band density.

### 4.7. Real-Time Quantitative Polymerase Chain Reaction (PCR)

After treatments, the total RNA of uterus and vagina was extracted with TRIzol reagent (Invitrogen, Carlsbad, CA, USA) according to the manufacturer’s instructions. The total RNA (2 μg) was reverse transcribed to cDNA using the High Capacity cDNA Reverse Transcription Kit (Applied Biosystems Foster City, CA, USA), according to the instructions manual. The specific transcripts were quantified by quantitative real-time PCR using the Quanti Tect SYBR Green PCR Kit (QIAGEN K.K., Tokyo, Japan) and analyzed with an ABI 7500 real-time PCR system (Applied Biosystems, Foster City, CA, USA). Gene-specific primers were used for ER α (forward: CGCCTTCTACAGGTCTAAT; reverse: GGTTCTTGTCAATGGTGC), ER β (forward: CTGTGAGGTAGGAATGCGAAAC; reverse: GGTCTGGGTGATTGCGAAGA) and β-action (forward: CCTCTATGCCAACACAGTGC; reverse: CTGTAGAACGGTGTGGTCATC). The mRNA levels of ER α and ER β were normalized to the β-action mRNA level. PCR was performed as 95 °C for 10 min, followed by 40 cycles of 95 °C for 30 s and 60 °C for 1 min. The quantification data was analyzed with ABI Prism analysis software. The relative mRNA expression was calculated with the comparative *C*_t_ method [28].

### 4.8. Statistics Analysis

The software, SPSS version 11.0 for Windows (SPSS Inc., Chicago, IL, USA), was used for statistical analysis. All data was expressed as the mean standard deviation and were analyzed by one-way analysis of variance (ANOVA) followed by least significant difference (LSD) or the Dunnett T3 test. Differences were considered statistically significant when the *p-*value was less than 0.05.

The article "Treatment with Panax Ginseng Antagonizes the Estrogen Decline in Ovariectomized Mice" was retracted in 2020. Reasons: duplicated images; concerns about the data.

## 5. Conclusions

This is the first report of estrogenic activity on reproductive tissues in OVX mice for ginseng. Ginseng is capable of restoring the estrus cycle, interfering with the atrophy of reproductive target tissues caused by ovariectomy. In addition, ginseng could relieve the symptoms of body weight gain induced by estrogen decline. These estrogenic effects may be mediated by stimulating the biosynthesis of estrogen in circulation and increasing the quantity of ERs in the target organs. This study also provides further evidence that ginseng can treat postmenopausal symptoms through action as an estrogen agonist.

## Figures and Tables

**Figure 1.** A chromatogram of the ginseng extracts. AU refers to absorbance unit.

**Figure 2.** The effect of ginseng (GS) on the estrous cycle. (**i**) Ovariectomized (OVX) mice untreated; (**ii**) Treated with estradiol valerate (EV) and (**iii**) Treated with ginseng (GS).

**Figure 3.** The effects of ginseng (GS) on body, uterine and adrenal gland weights. (**A**) Body weight was measured once a week for four weeks; (**B**) The weights of uterus and adrenal gland were measured at the end of the four-week treatment period. Data are the mean standard deviation (SD) of samples from 10 mice. *p-*values are for the one-way analysis of variance (one-way ANOVA) comparing the treatment group with untreated OVX mice. *** *p* < 0.001; ** *p* < 0.01; and * *p* < 0.05; compared with the OVX group. ^###^ *p* < 0.001; ^##^ *p* < 0.01; compared with the sham group. ^▲^ *p* < 0.05, compared with the EV group.

**Figure 4.** The effects of ginseng (GS) on serum estradiol (E_2_), luteinizing hormone (LH) and follicle-stimulating hormone (FSH) in OVX mice. Serum levels of E_2_ (**A**); LH (**B**) and FSH (**C**) were measured at the end of the treatment period. Data are the mean standard deviation (SD) of samples from 10 mice. *p-*values are for the one-way ANOVA comparing the treatment group with untreated OVX mice. *** *p* < 0.001; ** *p* < 0.01; compared with the OVX group. ^###^ *p* < 0.001; ^##^ *p* < 0.01; compared with the sham group.

**Figure 5.** The effects of ginseng (GS) treatment on the histology of uterus and vagina in the OVX mice. Representative photomicrographs taken at 200× magnification of uterus and 400× magnification of vagina sections from each treatment group are shown: (**i**) sham-operated mice; (**ii**) untreated ovariectomized (OVX) mice; (**iii**) OVX mice treated with estradiol valerate; (**iv**) OVX mice treated with GS at 12.0 g/kg; (**vi**) 18.0 g/kg (**v**) and 24.0 g/kg.

The article "Treatment with Panax Ginseng Antagonizes the Estrogen Decline in Ovariectomized Mice" was retracted in 2020. Reasons: duplicated images; concerns about the data.

**Figure 6.** The effects of ginseng (GS) treatment on the expressions of estrogen receptor (ER) α and (ER) β in the uterus and vagina. ER α and ER β expressions were assessed by quantitative immunohistochemistry. Representative photomicrographs taken at 400× magnification of uterus and vagina sections from each treatment group are shown: (**i**) sham-operated mice; (**ii**) untreated ovariectomized (OVX) mice; (**iii**) OVX mice treated with estradiol valerate; (**iv**) OVX mice treated with GS 12.0 g/kg; (**vi**) 18.0 g/kg (**v**) and 24.0 g/kg. Data are the mean standard deviation (SD) of samples from 10 mice. *p-*values are for the one-way ANOVA comparing the treatment group with untreated OVX mice. *** *p* < 0.001; ** *p* < 0.01; and * *p* < 0.05; compared with the OVX group; ^###^ *p* < 0.001, compared with the sham group.

**Figure 7.** The effects of ginseng (GS) on the expressions of estrogen receptor (ER) α and ER β at protein levels (**A**) and mRNA levels (**B**) in uterus and vagina of mice. The methods of western blot analysis and real-time PCR analyses were carried out as described in the Materials and Methods. Representative blots are shown above, and quantitative analyses are shown below. Values given are the mean standard deviation (SD) of three independent experiments. *** *p* < 0.001; ** *p* < 0.01; and * *p* < 0.05; compared with the OVX group. ^###^ *p* < 0.001; and ^##^ *p* < 0.01; compared with the sham group.
